# Up-Regulation of MiR-300 Promotes Proliferation and Invasion of Osteosarcoma by Targeting BRD7

**DOI:** 10.1371/journal.pone.0127682

**Published:** 2015-05-26

**Authors:** Zhen Xue, Jindong Zhao, Liyuan Niu, Gang An, Yashan Guo, Linying Ni

**Affiliations:** 1 Department of Orthopaedic Surgery, The Affiliated No.2 Hospital of Harbin Medical University, Harbin, Heilongjiang Province, 150086, China; 2 Department of Orthopaedic Surgery, the Fifth Hospital of Harbin City, Harbin, Heilongjiang Province, 150040, China; 3 Department of Physical diagnosis, The Affiliated Hospital of Harbin Institute of Technology, Harbin, Heilongjiang Province, 150001, China; 4 Department of Orthopaedic Surgery, The Tumor Hospital of Harbin Medical University, Harbin, Heilongjiang Province, 150086, China; Peking Union Medical College Hospital, CHINA

## Abstract

Increasing reports suggest that deregulated microRNAs (miRNAs) might provide novel therapeutic targets for cancers. However, the expression and function of miR-300 in osteosarcoma is still unknown. In our study, we found that the expression of miR-300 was up-regulated in osteosarcoma tissues and cells compared with paired adjacent non-tumor bone tissues and osteoblastic cells using RT-qPCR. The enforced expression of miR-300 could promote cell proliferation, invasion and epithelial-mesenchymal transition (EMT). Moreover, we identified that bromodomain-containing protein 7 (BRD7), a new tumor suppressor gene, was a direct target of miR-300. Ectopic expression of BRD7 could significantly inhibit miR-300-promoted proliferation, invasion and EMT. Therefore, our results identify an important role for miR-300 in osteosarcoma through regulating BRD7 expression.

## Introduction

Osteosarcoma is the most common primary bone malignancy with high local aggressiveness and rapid metastasizing potential, resulting in poor survival[1–3]. Despite current treatments combining chemotherapy, surgery, and sometimes radiotherapy, the 5-year cumulative survival rate of primary osteosarcoma wasonly 50%–60%[4–6]. Therefore, it is crucial to identify novel molecules and novel alternative therapeutic strategies to improve clinical outcome of patients suffering from osteosarcoma.

miRNAs (microRNAs) are a family of small, non-coding, endogenous RNAs (19–24 nucleotides in length), which inhibit gene expression by binding to the 3’untranslated region (3’-UTR) of mRNA sequence, leading to translational degradation or repression[7–12]. It has been demonstrated that miRNAs play crucial roles in cell biology such as cell proliferation, apoptosis, cell cycle, migration and invasion[13–19]. Increasing evidence shows the potential involvement of miRNAs in development in various human cancers such as gastric cancer, bladder cancer, lung cancer, hepatocellular carcinoma, and breast cancer[20–24]. miRNAs can function as either tumor suppressors or oncogenes according to their target genes[25, 26].

In this study, we showed the expression of miR-300 was increased in osteosarcoma tissues and cell lines compared with paired adjacent nontumor bone tissues and osteoblastic cells. Overexpression of miR-300 promoted cell proliferation and invasion and induce EMT. Moreover, we revealed that bromodomain-containing protein 7 (BRD7) was a direct target of miR-300 in osteosarcoma cells.

## Materials and Methods

### Ethics Statement

All of these patients (or patients’ parents on behalf of the children) agreed to participate in the study and gave written informed consent. Both this study and consent were approved by the Ethics Committee of The Second Affiliated Hospital of Harbin Medical University and complied with the Declaration of Helsinki.

### Cell lines and samples

Osteosarcoma cell lines MG63, U2-OS, Saos-2, and HOS and immortalized human fetal osteoblastic cell line hFOB 1.19 were obtained from the American Type Culture Collection (ATCC, Rockville, MD, USA) and were cultured in RPMI-1640 medium supplemented with 10% fetal bovine serum (GIBCO, NY, USA). Human osteosarcoma tissues and adjacent normal bone tissues were obtained from routine therapeutic surgery in our Hospital.

### Oligonucleotides and Cell Transfection

The miR-300 mimics and scrambled were purchased by GenePharma (Shanghai, China). For the transfection experiment, a complex of 20nM microRNAs and Lipofectamine 2000 (Invitrogen, CA, USA) mentioned above was prepared according to manufacturer’s instructions.

### Real-time quantitative PCR

Total RNA from tissues or cells was harvested using Trizol reagent (Invitrogen, Calsbad, CA, USA). The expression of miRNAs was detected using Taqman MicroRNA Assay (Applied Biosystems) according to manufacturer’s instruction. Quantitative real-time PCR was performed on the Applied Biosystems 7500 Real-Time PCR systems and using a TaqMan Universal PCR Master Mix. U6 snRNA was used as an internal control to miRNA expression. The expression of mRNA was normalized to GAPDH. (S1 Table)

### Cell Proliferation Assay

Cells were incubated in 10% CCK-8 (Dojindo, Kumamoto, Japan) diluted in medium until visual color conversion occurred. Proliferation rates were detected at 0, 12, 24, 48 and 72h after transfection.

### Western Blot Analysis

Total proteins were isolated from tissues or cells. Proteins were separated by 10% SDS-PAGE, transferred to NC membrane (Amersham Bioscience, Buckinghamshire, UK). After blocking with 10% nonfat milk for 2 h, membranes were immunoblotted with antibodies overnight, followed by HRP-linked secondary antibodies (Santa Cruz, USA). Protein levels of GAPDH were used as loading controls.

### Invasion analysis

Invasion assays were performed using Transwell invasion chambers coated with Matrigel (BD, USA) according to manufacturer’s instruction. Cells were transfected with miR-300 mimic or scramble and transferred on the top of Matrigel-coated invasion chambers in a serum-free DMEM. 10% fetal calf serum was added to the lower chambers. After 24 h, cells that remained on the top of the filter were wiping off and cells that migrated to the lower surface were stained with 0.2% crystal violet solution (Sigma) and counted.

### Luciferase assay

Cells were co-transfected with firefly luciferase reporter vector containing the BRD7 3’-UTR or its 3’-UTR mutant and the control vector containing Renilla luciferase, pRL-TK (Promega), in a final volume of 0.5 ml performed with lipofectamine 2000 (Invitrogen). Firefly and Renilla luciferase activities were detected using dual luciferase assays (Promega) after 48 hours transfection[27].

### Statistical Analysis

Statistical analyses were done using SPSS 17.0. Data are presented as the mean ± standard deviation. Statistical analyses were performed with either an analysis of variance (ANOVA) or Student’s t-test, and the statistical significance level was set at α = 0.05 (two-side). Each experiment was repeated at least three times.

## Result

### The expression of miR-300 was up-regulated in osteosarcoma

RT-qPCR analysis showed that miR-300 level was higher in four osteosarcoma cell lines, namely, MG63, U2-OS, Saos-2, and HOS, than in the osteoblastic hFOB1.19 cell line (Fig 1A). The expression of miR-300 in osteosarcoma tissues was up-regulated in 75% cases compared with corresponding adjacent normal tissues (Fig 1B). The level of miR-300 was higher in osteosarcoma tissue than in normal tissues in the 20 pairs (Fig 1C).

**Fig 1:** The expression of miR-300 was up-regulated in osteosarcoma. (A) The expression of miR-300 was detected in osteosarcoma cell lines (MG63, U2-OS, Saos-2 and HOS)and the osteoblastic hFOB1.19 cell line usingqRT-PCR analysis. (B) qRT-PCR analysis of miR-300 expression in 20 pair’sosteosarcoma tissues and their corresponding adjacent normal tissues. (C) Relative miR-300expressionlevels inosteosarcoma tissues and their corresponding adjacent normal tissues.***p<0.001.

### Over-expression of miR-300 promoted cell growth and invasion

miR-300 were over-expressed in MG-63 cells transfected with miR-300 mimics (Fig 2A). Overexpression of miR-300 promoted MG-63 cells proliferation (Fig 2B). Moreover, invasion analysis showed that mimics transfection increased the MG-63 cells invasion (Fig 2C).

**Fig 2:** Over-expression of miR-300 promoted cell growth and invasion. (A) qRT-PCR analysis of miR-300 expression after the transfection of miR-300 mimics or scramble. (B)The CCK8 proliferation assay used to study the proliferation of theMG-63 cells after transfection with the miR-300 mimics or scramble or no transfection. (C) overexpression of miR-300 promoted the MG-63 cells invasion. The relative invasive cells were shown in the right. ** p<0.01, and ***p<0.001.

### Overexpression of miR-300 induces EMT

As measured by qRT-PCR, we showed that ectopic expression of miR-300 inhibited the E-cadherin expression and induce the expression of N-cadherin, Vimentin and PI3K (Fig 3A). As expected, up-regulation of miR-300 can repress the protein expression of E-cadherin and promote the protein expression of N-cadherin, Vimentin and PI3K (Fig 3B).

**Fig 3:** Overexpression of miR-300 induces EMT. (A) qRT-PCR analysis showed that ectopic expression of miR-300 can inhibit the E-cadherin expression and induce the expression of N-cadherin, Vimentin and PI3K. (B) Western blot analysis showed that up-regulation of miR-300 can repress the protein expression of E-cadherin and promote the protein expression of N-cadherin, Vimentin and PI3K.

### BRD7 is a direct target of miR-300 in osteosarcoma cells

We found that BRD7 was a putative target gene of miR-300 using database TargetScan (Fig 4A). To obtain further direct evidence that BRD7 was a target of miR-300, we characterized the binding site of miR-300 in the 3’UTR of BRD7 mRNA. The results showed that miR-300 but not scramble specifically decreased the luciferase activity (Fig 4B). The mutant reporter cotransfected with miR-300 did not show significant decrease in the relative luciferase activity. Overexpression of miR-300 reduced the protein level of BRD7 in MG-63 cells (Fig 4C).

**Fig 4:** BRD7 is a direct target gene of miR-300 in osteosarcoma cells. (A) The sequences of miR-300 binding sites within the human BRD7 3’UTRs and schematic reporter constructs, in this panel, BRD7-WT represent the reporter constructs containing the entire 3’UTR sequences of BRD7. BRD7-MUT represent the reporter constructs containing mutated nucleotides. (B) The analysis of the relative luciferase activities of BRD7-WT, BRD7-MUT. (C) Overexpression of miR-300 reduced the protein level of BRD7 in the MG-63 cells using Western blot.

### miR-300 promotes cell proliferation and invasion by targeting BRD7

CCK8 proliferation assay showed that restoration of BRD7 inhibited the MG-63 cells proliferation (Fig 5A). As measured by qRT-PCR and Western blot, overexpression of BRD7 up-regulated expression of epithelial biomarker, Ecadherin, and reduced expression of mesenchymal biomarker, N-cadherin and Vimentin and the expression of PI3K (Fig 5B and 5C). Furthermore, the invasion abilities of miR-300 overexpressing MG-63 cells were partially repressed after pCDNA-BRD7 transfection (Fig 5D).

**Fig 5:** miR-300 promotes cell proliferation and invasion by targeting BRD7. (A)CCK8 proliferation assay of growth in pCDNA-BRD7 transfected miR-300 overexpressing MG-63 cells. (B)qRT-PCR analysis of the mRNA expression of E-cadherin N-cadherin and Vimentin in pCDNA-BRD7 transfected miR-300 overexpressing MG-63 cells. (C) Western blot analysis of the protein expression ofE-cadherin N-cadherin and Vimentin in pCDNA-BRD7 transfected miR-300 overexpressing MG-63 cells. (D) Invasion analysis of the invasion abilities in pCDNA-BRD7 transfected miR-300 overexpressing MG-63 cells. The relative invasive cells were shown in the right. *p<0.05, and ***p<0.001.

## Discussion

The deregulated expression of miRNAs has been identified in many cancers and their aberrant expression has been reported to highly correlate with the progression and prognosis of cancers[16, 17, 28, 29]. In this study, we found that the expression of miR-300 was up-regulated in osteosarcoma tissues and cell lines compared with paired adjacent non-tumor bone tissues and osteoblastic cells. Forced expression of miR-300promoted cell proliferation and invasion and induced EMT. Moreover, we revealed that BRD7 was a direct target of miR-300 in osteosarcoma cells. We demonstrated that miR-300 promoted cell proliferation and invasion by targeting BRD7. These results suggest that miR-300 may play a crucial role in regulating osteosarcoma cell proliferation and invasion through suppression of BRD7.

Previous studies have reported that miR-300 could act as an oncogene or a tumor suppressor in different cancers, dependent on cellular context[30, 31]. The expression of miR-300 was upregulated in glioma tissues and glioma stem-like cells (GSLCs). Overexpression of miR-300 promoted the self-renewal, proliferation of GSLCs and reduced their differentiation toward both astrocyte and neuronal fates[30]. However, *Yu et al*.reported that miR-300 was down-regulated in the head and neck squamous cell carcinoma (HNSCC) cells and breast cancer cells[31]. Overexpression of miR-300 could block TGF-beta-induced EMT and reverse the phenotype of EMT in HN-12 and MDA-MB-231 cells. In our study, the expression of miR-300 was higher in osteosarcoma tissues and cell lines compared with paired adjacent non-tumor bone tissues and osteoblastic cells. Moreover, overexpression of miR-300 promoted cell proliferation and invasion and induce EMT. These results imply that miR-300 may function as an oncogene in osteosarcoma.

Our results revealed that BRD7 was a direct target of miR-300 in osteosarcoma. BRD7, a member of the bromodomain-containing proteins family, was ubiquitously expressed in human tissues, including brain, heart, lung, colon and breast[32]. Previous evidences reported that BRD7 was localized predominently in the nucleus using immunofluorescence experiments and could bind to acetylated histone H3, and therefore regulate chromatin remodeling[33–35]. Increasing studies revealed that BRD7 might serve as a tumor suppressor gene in various tumors[36–38]. For example, the expressionof BRD7 was downregulated in colorectal carcinoma and nasopharyngeal carcinoma[39, 40]. Moreover, overexpression of BRD7 could inhibit nasopharyngeal carcinoma cell proliferation through multiple mechanisms, such as cell cycle arrest by transcriptionally regulating ras/MEK/ERK, Rb/E2F, b-catenin and ERK pathways[40]. Another study showed that BRD7 could inhibit prostate cancer cells proliferation by decreasing the transcriptional activity of androgen receptor (AR) up-regulated by tripartite motif (TRIM) proteins[41]. Furthermore, knocking down BRD7 allows p85α to accumulate in the cytosol and stabilize p110 levels and thereby enhance PI3K signaling[42, 43]. Here, BRD7 was identified as an important downstream target of miR-300. miR-300 directly bound to the 3’-UTR of BRD7, which contained a miR-300-binding site using a dual-luciferase reporter assay. Up-regulation of miR-300 significantly reduced the BRD7 protein level in osteosarcoma cells, and the inhibitory effects of miR-300 overexpression on osteosarcoma cell proliferation and invasion were reversed by upregulation of BRD7. Together, these data suggest that miR-300 might inhibit osteosarcoma proliferation and metastasis through regulating BRD7.

In conclusion, the present study demonstrated that miR-300 was increased in osteosarcoma tissues and cell lines. Overexpression of miR-300 promoted the cell proliferation, invasion and EMT of osteosarcoma through targeting BRD7. To the best of our knowledge, this is the first study to demonstrate that the miR-300/BRD7 axis regulates the proliferation, invasion and EMT of osteosarcoma cells. Repressed miR-300 expression might lead to the increased expression of BRD7 and in turn inhibit the progression of osteosarcoma.

## Supporting Information

S1 Table Primer sequence. (DOCX)
